This article has been retracted.

# Gastroprotective activity of a novel Schiff base derived dibromo substituted compound against ethanol-induced acute gastric lesions in rats

**DOI:** 10.1186/s40360-019-0292-z

**Published:** 2019-02-15

**Authors:** Kamelia Saremi, Sima Kianpour Rad, Faezeh Tayeby, Mahmood A. Abdulla, Hamed Karimian, Nazia Abdul Majid

**Affiliations:** 1 Institute of Biological Science, Faculty of Science, University of Malaya, 50603 Kuala Lumpur, Malaysia; 2 Department of Molecular Medicine, Faculty of Medicine, University of Malaya, 50603 Kuala Lumpur, Malaysia; 3 Department of Biomedical Science, Faculty of Medicine, University of Malaya, 50603 Kuala Lumpur, Malaysia; 4 School of Medicine, Faculty of Health & Medical Sciences, Taylor’s University, 47500 Subang Jaya, Malaysia

**Keywords:** Anti gastric ulcer, Schiff base compounds, Antioxidant enzymes, HSP70 protein

## Abstract

**Background:**

Basic function of bromine in body is to activate pepsin production in gastritis with low acidity. The present study encompasses a broad in vivo study to evaluate gastroprotective activity of a novel dibromo substituted Schiff base complex against Sprague Dawley (SD) rats.

**Methods:**

2, 2′-[1, 2-cyclohexanediylbis (nitriloethylidyne)]bis(4-bromophenol) (CNBP) is synthesized via a Schiff base reaction, using the related ketone and diamine as the starting materials. SD rats are divided as normal, ulcer control (5 ml/kg of 10% Tween 20), testing (10 and 20 mg/kg of CNBP) and reference groups (omeprazole 20 mg/kg). Except for the normal group, the rest of the groups are induced gastric ulcer by ethanol 1 h after the pre-treatment. Ulcer area, gastric wall mucus, and acidity of gastric content of the animal stomachs are measured after euthanization. Antioxidant activity of the compound is tested by Ferric reducing antioxidant power (FRAP) test and safety of the compound is identified through acute toxicity by [3-(4,5-dimethylthiazol-2-yl)-2,5-diphenyltetrazolium bromide (MTT) assay. Moreover, activities of superoxide dismutase (SOD), catalase (CAT), levels of prostaglandins E_2_ (PGE_2_) and also malondialdehyde (MDA) are determined.

**Results:**

Antioxidant activity of CNBP was approved via FRAP assay. Vast shallow hemorrhagic injury of gastric glandular mucosa was observed in the ulcer group compared to the CNBP-treated animals. Histological evaluations confirmed stomach epithelial defense effect of CNBP with drastic decrease of gastric ulceration, edema and leucocytes penetration of submucosal stratum. Immunostaining exhibited over-expression in HSP70 protein in CNBP-treated groups compared to that of the ulcer group. Also, gastric protein analysis showed low levels of MDA, PGE_2_ and high activity of SOD and CAT.

**Conclusions:**

CNBP with noticeable antioxidant property showed gastroprotective activity in the testing rodents via alteration of HSP70 protein expression. Also, antioxidant enzyme activities which were changed after treatment with CNBP in the animals could be elucidated as its gastroprotective properties.

## Background

Some aggressive factors, such as stress, alcohol or long term anti-inflammatory drugs consumption can develop lesions in stomach and provide suitable conditions for provoking peptic ulcer. In general, gastrointestinal ulcer involves injury in lining of stomach, causing destruction of muscularis and gastrointestinal tract mucosa [1].

Internal aggressive factors, such as pepsin, hydrochloric acid or refluxed bile, attack protective elements, e.g. bicarbonate mucus barrier, causing higher chance for developing gastrointestinal ulcer [2].

Some chemical compounds, such as phenolic, flavonoids, metallic and nonmetallic organic derivatives and heterocycles, Schiff bases, etc., possess anti gastric ulcer activity [3, 4]. Schiff bases are synthesized by reaction of primary amines with carbonyl compounds [5]. Chelation of such compounds with some metals [6–8], halogens [9, 10], oxygen [11], etc. demonstrated to have applications as drugs and possess many biological activities, such as, anti-viral [4], anti-bacteria [11], gastroprotective activity [12], antioxidant [13], anti-inflammation [14] and anti-tumors [15]. Specifically, it is noted that bromine substituted complex of Schiff bases exhibits excellent activity against gastro ulcer in rodents [16]. Basic functions of bromine in body include activity in digestion of carbohydrates and fats and also enhancing pepsin production in gastritis with low acidity [17, 18].

### Objective

The present study demonstrates synthesize of a novel chemical compound (CNBP) and study of its antioxidant and gastro protective activity in rodent by analyzing effect of the compound on antioxidant enzymes activity.

## Materials

### Drugs

All the necessary chemicals for the syntheses were purchased from Merck and Sigma-Aldrich chemical companies. SD rats were obtained from the Animal Experimental Unit (AEU), Faculty of Medicine, University of Malaya. Paraffin tissue processing equipment, ketamine and xylazine for anesthetizing the animals and tween 20 were purchased from Sigma-Aldrich, Germany. Omeprazole was obtained from TROGE Medical GMBH, Germany. Sucrose, magnesium chloride and alcian blue, MTT reagent, thiazolyl blue and tetrazolium bromide were all purchased from USB Affymetrix.

## Methods

### Synthesis and characterizations of CNBP

The Schiff base derivative, entitled: 2, 2′-[1, 2-cyclohexanediylbis(nitriloethylidyne)]bis(4-bromophenol) (CNBP) was prepared via the following protocol [19]: A solution of trans-1,2-diaminocyclohexane (2.5 g, 21.9 mmol) in methanol (70 ml) was reacted with 5-bromo-2-hydroxyacetophenone (9.42 g, 43.8 mmol) in presence of catalytic amount of acetic acid under reflux condition for 6 h. After cooling to ambient temperature, a yellowish green solid was formed via filtering, washed with methanol and finally dried over phosphorus pentoxide (Fig. 1). It was recrystallized from ethanol to afford CNBP (8.45 g, 76%), m.p. 220–222 °C.

**Fig. 1:** Synthesis of the Schiff base (2)

IR [KBr]: 3500 cm^− 1^ (OH), 3020 cm^− 1^ (CH_aromatic_), 2940, 2860 cm^− 1^ (CH_aliphatic_), 1605 cm^− 1^ (C=N), 1560 cm^− 1^(C=C), 1256 cm^− 1^(C-N); ^1^H NMR (400 MHz, CDCl_3_): *δ* 7.60/(7.48) (d, 2H, ^3^*J* = 2.4 Hz, 2x Ar-H), 7.30/(7.29) (dd, 2H, ^3^*J* = 8.9 Hz, 2x Ar-H), 6.77/(6.75) (d, 2H, ^3^*J* = 8.9 Hz, 2x Ar-H), 4.60/(3.85) (m_c_, 2H, 2x CH-N), 2.32/(2.25) (s, 6H, 2x CH_3_), 1.9 (t~m_c_, 4H, 2x CH_2_-CH), 1.79–1.57 (m_c_, 2H, CH_2_), 1.48 (p~m_c_, 2H, CH_2_).^13^C NMR (100 MHz, CDCl_3_): *δ* 170.16 (169.95) 2x (C=N), (163.01) 162.83 2x (Ar-OH), 135.24 (135.16), 130.87 (130.70) 2x (CH_Ar_) 120.82 (120.78) 2x (C_Ar_-CN) 120.62 (120.51) 2x (CH_Ar_), 108.79 (108.57) 2x (Ar-Br), 63.21 (59.61) 2x (CH-N), 32.33 (29.81), 24.19 (22.29) 2x (CH_2_CH_2_), 14.57 (14.52) 2x (CH_3_).

### Cytotoxicity activity

#### MTT cytotoxicity assay

An acute toxicity test, MTT, was done on fibroblast cells (BJ-5ta) to find a safe dose of the compound. Fibroblast cells were cultured in DMEM medium and enriched with 110 mg sodium pyruvate/L, 4500 mg glucose/L, L-glutamine, 10% FBS and 1% antibiotics (penicillin and streptomycin). It was then incubated at 37 °C in 5% CO_2_ in a humidified AIR Jacketed incubator (AutoFlow NU-4750 Water Jacket CO2 Incubator). 0.5 × 10^5^ cells/ml was seeded into a 96-well plate followed by overnight incubation. Different doses of CNBP (100, 50, 25, 12.5 and 6.25 μg/ml) 100 μl were diluted in distilled water, control with 0.25% of DMSO added into each well. After 48 h incubation, 20 μl of MTT solution was added to each well and followed by addition of 100 μl of DMSO and the absorbance was read by a plate reader (Tecan, The Infinite M200, Mannedorf, Switzerland) at 570 nm [19]. The percentage of growth of the cells under influence of the compound was calculated by the following formula:

$$ \%\mathrm{cell}\ \mathrm{viability}=\kern0.37em \left(\mathrm{Abs}\ \mathrm{of}\ \mathrm{compound}\div \mathrm{Abs}\ \mathrm{of}\ \mathrm{control}\right)\times 100 $$

### Ferric reducing antioxidant power (FRAP) test

Reduction of ferric tripyridyl triazine (Fe III TPTZ) complex to its ferrous form (intense blue color) at low pH can be monitored by measuring the absorbance change at 593 nm (0 and 4 min). 300 mmol/l sodium acetate buffer (pH 3.6) and ferric chloride were added (20 mM) to the complex followed by addition of tripyridyl triazine (TPTZ; 0.0625 g in 40 mM HCl). For preparation of FRAP reagent, the above reagents were mixed in a ratio of 10:1:1. CNBP (10 μl) was added to 300 μl of FRAP reagent and gallic acid and ascorbic acid were used as the controls.

### Experimental animals and ethical statement

Forty-eight healthy SD rats (6–8 weeks old, 200–250 g) were housed in plastic cages under standardized environment (23 ± 2 °C, 12 h light/ 12 h dark cycle) and permitted freely to water, *libitum* and standard chow pellets. The rats were acclimatized to laboratory condition for 1 day prior to experiments without any access to food. The experimental processes including the protocols in this study were approved by the Ethics Committee of the Research Centre and in accordance with the recommendations of the University of Malaya; Council on Animal Care Guidelines for the proper care and use of laboratory animals (Ethic no. 2015-09-11/BMS/R/MAA).

### Study design and experimental procedure

Eighteen female rats were divided into three equal groups, namely, the control group was administrated orally with 5 ml 10% Tween 20, and the tested groups were administrated with low dose (100 mg/kg; LD) and high dose (200 mg/kg dose; HD) of CNBP, respectively. The animals were accessed to food but not water overnight and at the end of the fasting period, it was followed by testing toxicity of the compound at 30 min, 2, 4, 24 and 48 h after the administration. The rats’ behavior changes were monitored and the rates of mortality were recorded after 14 days [20, 21]. The testing animals were then euthanized with ketamine (30 mg/kg) and xylazine (3 mg/kg) and the blood samples were collected via cardiac puncture for serum biochemistry analyzing. The liver and kidney were used for the histopathology and immunochemistry evaluation [22].

### Gastric ulcer induction by ethanol

The rats were divided into five groups, six rats in each. After an overnight fast (food but not water), normal and ulcer control groups received 5 ml/kg of 10% Tween 20. The reference group was given 20 mg/kg omeprazole in the volume of 5 ml/kg, and the experimental groups were administrated with low and high doses of CNBP (10 and 20 mg/kg). All the treatments were fed to the rats via oral gavage. After 1 h, in order to induce stomach injury, the other five groups, except the normal group were exposed to oral gavage of absolute alcohol. After additional hour, the rats were sacrificed followed by removing their stomachs, immediately for carrying out the further tests [21, 23].

### Assessment of gastric fluid acidity

The stomachs were opened along the greater curvature and the juices were collected in the separate labeled tubes. The contents of each stomach was centrifuged at 3000 rpm for 10 min and the supernatant was assessed for pH measurement via digital pH meter titration, using 0.1 NaOH solution [24].

### Determination of gastric wall mucus (GWM)

Stomach epithelia’s mucus assay was carried out according to the method conducted by Corne et al. [25]. The glandular segments of each stomach were removed, weighed, and transferred immediately to 10 ml of 0.1% *w*/*v* Alcian blue solution containing 0.16 M sucrose solution buffered with sodium acetate (0.05 M pH 5) for 2 h immersion. The excess dye in each segment was removed using 10 ml of 0.25 M of sucrose and the rest was washed out by 10 ml of 0.5 M of magnesium chloride for 30 min. The remained tissue was removed and mixed up with 4 ml ethyl ether and was shaken for 2 min, centrifuged at 3000 rpm for 10 min. The absorbance of the supernatant was measured at 598 nm. The exact amount of Alcian blue which was extracted of the glandular stomach tissues were calculated via the formula which was suggested by Piper [20].

### Measurement of the ulcer area

The length and width (mm) of each hemorrhagic lesion were measured using a pelanimeter (10 × 10 mm^2^  =  ulcer area) individually under a dissecting microscope with a magnification of 1.8x. The sum of the area of the lesions for every stomach was used to calculate the ulcer area (UA) [26]. The UI was calculated using the following formula [27]:

$$ {\displaystyle \begin{array}{l}\left(\mathrm{UI}\%\right)=\left[\left(\mathrm{UA}\ \mathrm{of}\ \mathrm{negative}\ \mathrm{control}-\mathrm{UA}\ \mathrm{of}\ \mathrm{treated}\right)\right./\left.\mathrm{UA}\ \mathrm{of}\ \mathrm{negative}\ \mathrm{control}\right]\times 100\\ {}\mathrm{UI}=\mathrm{Ulcer}\ \mathrm{Inhibition}\end{array}} $$

### Antioxidant activity

#### Gastric homogenate preparation

Tissue homogenization was carried out according to a study conducted by Sidahmad et al. [28]. A small piece of glandular segments of each stomach was homogenized by ice-cold 50 mM PBS (4 °C pH 7.2), containing mammalian protease inhibitor cocktail, using Teflon homogenizer (Polytron, Heidolph RZR 1, Germany) following by centrifuging the resulting tissues (15 min, 4500 rpm).

#### Measurement of stomach’s protein concentration

Protein concentration measurements was carried out for the homogenate stomach tissues (1 mg/ml) using Biuret reaction [29].

#### Superoxide dismutase (SOD) activity assay

The activity of gastric SOD was evaluated using Superoxide Dismutase Assay kit from Cayman Chemicals (USA). This assay was carried out based on the instruction provided by the manufacturer. SOD activity was expressed as U/ml, where one unit is defined as the amount of enzyme needed to exhibit 50% dismutation of the superoxide radicals.10 μl of the sample was mixed with 200 μl of diluted radical detector in 96-well plate and the reaction was started by adding 20 μl of diluted xanthine oxidase and after 20 min of incubation, the absorbance was read at 440–460 nm.

#### Catalase (CAT) activity assay

The activity of the gastric’s CAT was evaluated using the Catalase Assay kit from Cayman Chemicals. 20 μl of the samples was mixed with 20 μl of catalase followed by addition of 20 μl of dilute hydrogen perioxide to start the reaction. After 20 min incubation, the reaction was terminated by adding 30 μl of diluted potassium hydroxide at room temperature for 10 min. 10 μl of catalase potassium periodate was added to the samples and left for another 5 min incubation, before reading the absorbance at 540 nm. The base of the assay is the reaction of CAT with methanol leading to production of H_2_O_2_ formaldehyde which is measured colorimetrically using 4-amino-3-hydrazino-5-mercapto-1, 2, 4-triazol (purpald) as the chromogen. CAT activity was expressed in nmol/min/ml, which one of the units is defined as the amount of enzyme that causes formation of 1.0 nmol of formaldehyde at 25 °C per min.

#### Membrane lipids peroxidation (MDA) level assessment

Malondialdehyde **(**TBARS) Assay kit from Cayman was used to measure MDA levels (mmol/g protein). 100 μl was pipetted from each sample and mixed with 100 μl of SDS solution and 4 ml of the color reagent. The samples were kept in a water bath at 100 °C for 1 h, followed by immediate transferring to ice bath to halt the reaction for 10 min. It was then centrifuged at 1600×g and 4 °C and the absorbance was read at 532 nm.

#### Prostaglandin E2 (PGE2) level assay

The level of gastric PGE2 was assayed using Prostaglandin Immunoassay kit (Uscn Life Science, China). The PGE_2_ was measured in pre-coated 96-well plate with the antibody which was specific for rat’s PGE_2_. The gastric PGE_2_ level was interpolated from the standard curve of the serially diluted stock solution (300 pg/ml) and the absorbance was read at 450 nm.

### Histology of gastric epithelium

#### Routine hematoxylin and eosin staining

Specimens of the stomach’s walls were fixed in 10% phosphate buffered formalin at room temperature and then processed in tissue-processing machine (dehydration, clearance and infiltration with paraffin) (Leica, Germany), followed by paraffin-embedded. The stomach tissues were sectioned at thickness of 5 μ, and then stained with hematoxylin and eosin for histological evaluation [30].

#### Evaluation of gastric mucosal glycoproteins

To observe gastric epithelial mucus secretion and also to evaluate alteration in either acidic or basic glycoproteins, the sections of the stomach’s walls (glandular portion) were stained with Periodic Schiff Base (PAS) stain [31].

### Evaluation of immunohistochemically stain of HSP70

Immunostaining of heat shock protein HSP70 protein was done according to the manufacturer’s protocol instruction of Dako kits (Dako Cyomation, USA).

## Experimental outcomes

It is found that CNBP shows antioxidant activity via FRAP test. The ulcer group has shown huge shallow hemorrhagic injury of gastric glandular mucosa compared to those animals which were pre-fed with CNBP. Histological analysis illustrated stomach epithelial defense effect of CNBP because of it’s remarkable decline of gastric ulceration, edema and leucocytes penetration of submucosal stratum. Immunostaining exhibited over-expression of HSP70 in CNBP-treated groups. Also, gastric protein indicated low levels of MDA and PGE_2_ and high activity of SOD and CAT.

## Statistical methods

All data are accessible as mean ± SEM. Differences among the experimental groups were determined by one-way ANOVA followed by Tukey’s post-hoc test for multiple comparisons using SPSS version 24. Values of *p* < 0.05 were considered as significant.

## Results

### CNBP has no cytotoxicity effect

The MTT assay was done to find out cytotoxicity effect of CNBP prior it’s evaluation of gastro protective activity on human cell lines. The effect of CNBP on fibroblast cell proliferation is depicted in Fig. 2. It was noticed that the cell viability was enhanced after treatment with CNBP which shows that it could affect the proliferation on the fibroblast skin cell. The threshold concentration for significant increase of cell proliferation was noticed at 6.2–12.5 μg/ml.

**Fig. 2:** Comparison of the effect of CNBP compound on fibroblast cell viability. The data (in triplicate) are represented as the mean ± SEM. **p < 0.01 with the untreated cells (control)

### Antioxidant properties of CNBP evaluated by FRAP assay

Power of CNBP in reducing ferric tripyridyl (Fe^+ 3^) to ferrous form (Fe^+ 2^), was found to be significant (Fig. 3). However, it’s FRAP value (628.8 ± 19.33 μmol Fe (II)/g), in comparison with ascorbic acid (973.7 ± 3.48 μmol Fe (II)/g) and gallic acid (2373.8 ± 84.70 μmol Fe (II)/g, is significantly lower.

**Fig. 3:** Comparison of the FRAP value of CNBP with the synthetic reference standard (ascorbic acid and gallic acid). The data are in triplicate and represented as the mean ± SEM. Significant differences are considered as ***P < 0.001. (# with ascorbic acid and $ with gallic acid)

### Evaluation of acute toxicity

The effect of CNBP on renal or liver function and lipids profiles of the rats is listed in Tables 1, 2, 3. The treated animals showed neither mortality nor signs of toxicity which was tested via renal, liver functions changes and lipids profiles analysis compared to the vehicle group. In addition, there were no histological changes in liver and kidney sections of all the groups during the time of experiment (Fig. 4).

**Table 1:** Effects of 100 mg/kg and 200 mg/kg of CNBP on Renal functions of SD rats (*n* = 6)

Animals group	Renal function test						
	Sodium (mM/l)	Pottasium (mM/l)	Chloride (mM/l)	CO_2_ (mM/l)	Anion (mM/l)	Urea (mM/l)	Creatinine (μM/L)
Control (10% Tween 20)	144.33 ± 0.27	4.43 ± 0.10	104.33 ± 0.27	24.00 ± 0.47	17.67 ± 0.54	6.73 ± 0.30	34.33 ± 0.54
CNBP(100 mg/kg)	141.67 ± 0.54	5.10 ± 0.33	104.67 ± 1.52	27.67 ± 1.09	14.33 ± 1.36	7.30 ± 0.29	38.67 ± 0.72
CNBP (200 mg/kg)	141.00 ± 0.47	5.63 ± 0.19	103.33 ± 0.98	28.33 ± 1.09	15.67 ± 0.27	6.50 ± 0.60	36.33 ± 1.91

**Table 2:** Effects of 100 mg/kg and 200 mg/kg of CNBP on Liver functions of SD rats (*n* = 6)

Animal groups	Liver function test								
	Total protein (g/l)	Albumin (g/l)	Globulin (g/l)	TB (μM/l)	CB (μM/l)	AP (IU/l)	ALT (IU/l)	AST (IU/L)	GGT (IU/L)
Control (10% Tween 20)	60.33 ± 0.27	40.33 ± 0.27	22.00 ± .0.47	1.83 ± 0.14	0.90 ± 0.15	119.00 ± 2.94	53.67 ± 1.19	126.67 ± 2.13	1.00 ± 0.00
CNBP(100 mg/kg)	59.33 ± 0.72	37.33 ± 0.54	22.00 ± 0.47	2.00 ± 0.00	0.95 ± 0.19	137.67 ± 0.27	54.67 ± 1.09	122.33 ± 3.60	1.67 ± 0.02
CNBP(200 mg/kg)	60.33 ± 1.36	38.67 ± 1.19	21.67 ± 0.54	2.00 ± 0.00	0.89 ± 0.21	143.00 ± 3.68	68.33 ± 3.31	151.00 ± 0.82	1.67 ± 0.27

*TB* Total bilirubin, *CB* Conjugated bilirubin, *AP* Alkaline phosphatase, *ALT* Alanine transaminase, *AST* Aspartate transaminase, *GGT* G-Glutaml transferase

**Table 3:** Effects of 100 mg/kg and 200 mg/kg of CNBP on Lipids profiles of SD rats (*n* = 6)

Animal groups	Lipid profile analysis			
	Triglyceride (mM/l)	Total cholesterol (mM/l)	HDL Cholesterol (mM/l)	LDL Cholesterol (mM/l)
Control (10% Tween 20)	0.40 ± 0.00	1.27 ± 0.07	0.40 ± 0.01	0.52 ± 0.04
CNBP(100 mg/kg)	0.30 ± 0.00	1.34 ± 0.05	0.46 ± 0.01	0.86 ± 0.04
CNBP(200 mg/kg)	0.33 ± 0.03	1.30 ± 0.09	0.41 ± 0.04	0.75 ± 0.05

The values are listed as mean ± S.E.M (*n* = 6). There were no significant differences (*P* < 0.05) between the groups

**Fig. 4:** Histological sections of kidney and liver (First & second row, respectively) (*n* = 6). **a** Vehicle control (10% Tween 20), **b** treated with CNBP (100 mg/kg) and **c** CNBP (200 mg/kg). No structural dissimilarity was detected among the treated and control group

### Effect of CNBP on the pH of gastric secretion and gastric wall mucus

Based on the method of in vivo confocal microscopy, it was initially necessary to make sure the stability of the animal preparation. Body temperature was measured with rectal thermistor probe in another series of nine animals before (36.0 ± 0.5 °C) and after (35.7 ± 0.2 °C) 3 to 4 h on the confocal stage. Both measurements indicated that the surgical preparation was stable. The pH values were found to be significantly (*P < 0.05* and *P < 0.001*) higher in the treated groups (*n* = 6) when compared to that of the ulcer group (Fig. 5). Pre-feeding of the treated rats with CNBP (HD) (*n* = 6), significantly increased GWM compared with that of the ulcerated group (*n* = 6) (Fig. 5).

**Fig. 5:** Effect of CNBP on the pH and GWM. Data are presented as Mean ± S.E.M (*n* = 6). Significant differences are considered as *P < 0.05 and ***P < 0.001. Reference group received 20 mg/kg omeprazole, low dose (LD) CNBP and high dose (HD) of CNBP

### Effect of CNBP on stomach mucosa

Gross features of those stomachs which were treated with CNBP (HD) (*n* = 6) showed significant reduction of acute ulcerated reddish and inflamed bands compared to the ulcer group (*n* = 6) which was confirmed by the ulcer area and % inhibition measurements (Fig. 6). Although Fig. 7 shows that pre-fed groups with LD (*n* = 6) and HD (*n* = 6) of CNBP could clear the lower ulcer area compared to the reference group (*n* = 6), they, significantly reduce in the ulcer area and % inhibition compared to that of the ulcerated class (*n* = 6).

**Fig. 6:** Effect of CNBP on gross images of absolute ethanol-provoked gastric injury in rats (*n* = 6). **a** Normal control gastric epithelium (10% Tween 20). **b** Ulcerated control (absolute ethanol) which exhibits extraordinary acute haemorrhagic ulceration (black arrow). **c** Reference control (omeprazole, 20 mg/kg) indicates mild injury, **d** & **e** Stomachs pre-fed with low dose of CNBP (LD) and high dose (HD), respectively show obvious reduction in the gastric lesions

**Fig. 7:** The ulcer area of CNBP. Significant differences are considered as ***P < 0.001 (*n* = 6). The rats which are pre-fed with CNBP significantly decreased the ulcer area when compared to ulcer control group. % ulcer inhibition of the reference and experimental groups are indicated above the bars

### Protein concentration in gastric homogenate

Pre-feeding of the animals with CNBP (*n* = 6) notably increased protein level of gastric homogenate in comparison with that of the ulcer control class (*n* = 6) (Table 4).

**Table 4:** Effect of the CNBP on the stomach homogenate endogenous antioxidant enzymes activities and, MDA and PGE_2_ levels, and protein concentration (*n* = 3)

Animal groups	SOD	CAT	MDA	PGE2	Protein concentration
	(U/mg protein)	(nmoL/min/mL protein)	(μmoL/g protein)	(ng/mg protein)	(mg/mL tissue)
10% Tween 20 (Normal control)	17.15 ± 0.90^***^ (*p*-value < 0.001)	82.51 ± 2.17^***^ (*p*-value < 0.001)	62.31 ± 2.90^***^ (*p*-value < 0.001)	3.08 ± 0.11^***^ (*p-*value < 0.001)	9.00 ± 0.11^***^ (*p*-value < 0.001)
Absolute EtOH (Ulcer control)	4.04 ± 0.33	18.70 ± 0.71	146.80 ± 3.53	1.01 ± 0.03	5.12 ± 0.40
Omeprazole (20 mg/kg)	20.07 ± 0.50^***^ (*p*-value < 0.001)	100.34 ± 0.56^***^ (*p*-value < 0.001)	82.64 ± 3.52^***^ (*p*-value < 0.001)	2.95 ± 0.06^***^ (*p*-value < 0.001)	7.71 ± 0.88^**^ (*p*-value = 0.003)
CNBP (LD)	12.22 ± 0.58^***^ (*p*-value < 0.001)	42.45 ± 2.48^*^ (*p*-value = 0.04)	112.48 ± 7.47^*^ (*p*-value = 0.04)	2.59 ± 0.24^***^ (*p*-value < 0.001)	6.03 ± 0.17 (*p*-value = 0.06)
CNBP (HD)	19.12 ± 1.14^***^ (*p*-value < 0.001)	68.30 ± 2.88^***^ (*p*-value < 0.001)	101.01 ± 7.67^**^ (*p*-value = 0.002)	2.88 ± 0.15^* **^ (*p*-value < 0.001)	6.72 ± 0.15^*^ (*p*-value = 0.04)

All values (in triplicate) are expressed as the mean ± SEM. significant at * *p* < 0.05, ** *p* < 0.01, and *** *p* < 0.001 compared to ulcerated group

### Gastric antioxidant activity

Ulcerated stomachs exhibited significant suppression in the endogenous antioxidant enzymes (SOD and CAT). In addition, the stomachs of the animal which were pre-fed with CNBP (*n* = 6), significantly enhanced the activities of SOD and CAT enzymes in comparison with the ulcer control class (*n* = 6) (Table 4). Based on the reference control group (*n* = 6) which were pre-fed with omeprazole (*n* = 6), either the low or high dose of CNBP showed low protein content of SOD and CAT (*p* < 0.05).

### MDA and PGE_2_ levels of gastric tissue homogenate

The animals which were pre-fed with CNBP (HD) (*n* = 6) showed significant attenuation in the gastric MDA level compared to the ulcer control group (*n* = 6) which were given absolute ethanol only. However, the gastric level of PGE_2_ indicated higher value in CNBP (HD)-pre-fed rats (*n* = 6) than that of the ulcer control (Table 4).

### Effect of CNBP on histological evaluation of gastric lesions

#### H & E staining

In the ulcer control group (*n* = 6), stomach wall showed drastic destruction of gastric mucosal surface with submucosal edema and significant inflammation. Those rats which were pre-fed with CNBP (HD) (*n* = 6) indicated remarkable gastric mucosal protection (Fig. 8).

**Fig. 8:** Effect of the CNBP on the histology of gastric epithelium in ethanol-provoked gastric mucosal damage in rats (*n* = 6). **a** Normal control rats. **b** Ulcer control stomach presenting severe mucosal injury (yellow arrow) along with deep necrosis (blue arrow), edema and inflammation of submucosal layer (black arrow). **c** Reference control stomach (omeprazole, 20 mg/kg) presenting mild mucosal injury. **d** & **e** experimental animals’ stomachs pre-fed with CNBP showing reduced mucosal damage, while the high dose of CNBP (**e**) showing better gastroprotective effect than the low dose (**d**)

#### PAS staining

Those rats which were pre-fed with CNBP (HD) (*n* = 6), showed drastic intense up-take of magenta color by the gastric epithelial glycoproteins. (*n* = 6) (Fig. 9).

**Fig. 9:** Effects of CNBP on PAS staining of gastric glycoproteins secretion of in ethanol-provoked stomach damage in rats (*n* = 6). **a** Normal control class indicating normal magenta color (black arrow) of gastric mucus glands. **b** Absence of PAS staining from the mucosa of ulcer control class exhibiting severe mucosal injuries. **c** Reference animals exhibiting intense PAS stain. **d** & **e** Tested groups were fed with the low dose (10 mg/kg) and high dose (20 mg/kg) of CNBP, respectively exhibited intense up-take of PAS stain. The high dose of CNBP is showing more intense PAS staining than the low dose (**d**)

### Effect of CNBP on immunohistochemically staining of gastric mucosal HSP70

The immunostaining of the gastric mucosa of the ulcer control group (*n* = 6), showed down-regulation of HSP70 protein. In the tested group, which was fed with CNBP (HD) (*n* = 6), showed up-regulation of HSP70 protein in their stomach tissues (Fig. 10).

**Fig. 10:** Effect of the CNBP on the expression of HSP70 protein of gastric mucosa in ethanol-induced stomach ulcer in rodents (*n* = 6). **a** Normal control group. **b** Ulcer control group expressed less HSP70 protein (yellow arrow). **c** Reference group demonstrated obvious up-regulation of HSP70 protein. **d** & **e** Tested groups pre-fed with CNBP (LD & HD) are exposing expression of HSP70 protein in the high dose group more effective than the low dose group

## Discussions

It was found that absolute ethanol could cause numerous adverse effects on epithelial cells, such as injury, which leads to depletion in various protein concentration [32]. Mucus membrane is known as the first layer of defense system in stomach tissues; therefore, when alcohol destroys it, variable irreparable losses are developed. Gastric mucosa as a barrier doesn’t permit digestion of enzymes, such as pepsin to diffuse into stomach wall [21]. Basically, mucus gel possess very low permeability to large molecules, such as pepsin, but some factors, like stress, alcohol, etc. can increase permeability which cause release of vasoactive products and finally vascular damages. Damaging vascular leads to necrotizing action in gastric cells, and as a result imbalances secretion of bicarbonate and production of mucus [23]. Furthermore, it is believed that generation of ROS caused by ethanol has significant role in ulcer formation [33].

Previous studies suggested close correlation between suppression of gastric acidity and effectiveness of treatment. Ability to attenuate gastric acid secretion is considered as mainstay of treatment for gastric ulceration [34]. It is well known that proton pump inhibitors drugs, such as omeprazole decreases the extra volume of acid which is produced in stomach. Such drugs are effective in acid-independent models, like ethanol-ulcer, exert mucosal protection and in non-anti-secretory doses [35]. Also, it is suggested that antioxidants, contain the ability of antigasteric ulcer [8, 16].

In the current study, pre-treatment with CNBP enhanced the generation of epithelial cells which gave rise to significant increase in protein concentration in the gastric secretions of the pre-treated groups.

Based on the previous studies, human fibroblast can be used for measuring the toxicity of compounds. In addition, this type of cell is studied when a new compound is supposed to be evaluated for its wound healing process [36, 37]. The acute toxicity properties of CNBP which was evaluated by MTT assay fibroblast cells (BJ-5ta) did not confirm any toxicity or mortality in the rats during the experiments. The test confirmed that CNBP is safe without toxicity when it was orally administered (100 and 200 mg/kg). Meanwhile, the FRAP assay indicated antioxidant activity of the testing compound in comparison with the controls (ascorbic acid and gallic acid). It is reported that certain antiulcer drugs increase amount of gastric mucus secretion in gastric mucus [27]. CNBP showed significant anti-ulcer activity in the rats, including contraction of the ulcer area, increment of pH and mucus weight, decrement of sub-mucosal edema and leukocyte infiltration. The outcomes of the present study were in accordance with some other studies which assessed the gastroprotective and anti-ulcer activity of different synthetic compounds [38, 39]. Pre-treatment with CNBP, significantly suppressed gastric acidity and also suppress the destruction of GWM in the rats treated with ethanol, indicating that the gastro protective effect of CNBP was mediated partially by preservation of the gastric wall mucus. Balance perturbation between gastro-protective mechanisms and gastrotoxicity of different agents is the basis of acute inflammation which could cause secretion of various inflammatory cytokines [40]. It is reported that acute inflammation induced by ethanol is accompanied by neutrophils infiltration of gastric wall mucus [21]. The current results demonstrated that submucosal infiltration was effectively suppressed by pre-treatment of the rats with CNBP compound. An extensive generation of ROS and free radicals cause metabolic impairments and irreversible cell damages in human body [41]. Gastric mucosal protection, inhibition of edema and inflammatory reactions of submucosal layer in the rats pre-treated with CNBP compound compared to the ulcer control group were reasserted by re-evaluation of the gastric tissues histologically [42].

Pre-treatment with CNBP, significantly increased the gastric mucus production and decreased the acidity of gastric content. The periodic acid-Schiff PAS staining results showed increase of the mucus production in the gastric walls of the rats pre-treated with CNBP which suggests the gastro-protective activity of the compound might be potentiality due to preservation of mucus secretion. These results were in agreement with several other studies that showed significant increase of gastric mucus in rats which were pre-treated with various synthetic compounds against necrotizing agent-induced gastric mucosal wounds [43].

ROS, such as superoxide radical anion is generated by neutrophils resulting in the reaction with cellular lipids and the production of lipid peroxides. Another effective indicator of oxidative stress which causes mucosal injuries could be MDA which is a major metabolite of lipid peroxidation [44]. Based on the study which was done by Hawkey & Rampton [45], PGE_2_ also plays a key role in regulation of gastric mucus secretion, hence, PGE_2_ possesses protective effects on different gastric injury in animal models studies [46]. It was reported that ethanol could decrease the content of mucosal PGE_2_ [47] exerting a protective action on the stomach through the activation of PGE_2_ receptors [48]. In addition, the mucosal level of PGE_2_ was increased in the experimental groups compared to the ulcer control class. Such enhancement in level of PGE_2_, suggests gastroprotective effect of CNBP which could be mediated, partially by PGE_2_.

Based on the current study, the oral administration of CNBP could protect against gastric ulceration by elevating SOD and CAT activities, and decreasing MDA and PGE_2_ levels. The results of this study are almost in line with the results which were reported by several researchers regarding that SOD and CAT activities were increased in synthetic compound-treated groups in comparison with ethanol-treated animals [42, 49, 50]. In addition, reduction in MDA levels were reported in the treated rats with several compounds, such as 3-(2-Chlorophenyl)-1-phenyl-propenone and Zn(II)–curcumin complex [51, 52]. It is reported that ROS, such as hydroxyl radicals, superoxide anions, and lipid peroxides are harmful species which is known to provoke gastric ulcer development [53]. Free radical ultimately causes depletion in tissue antioxidant status leading to lipid peroxidation. Hence, antioxidants scavenge free radical formation which play major role in protection of cellular damage. Treatment with CNBP enhanced the antioxidant enzymes levels/activities compared to the ulcer group preventing free radical generation which could happen during ulcer development.

Hsp70 is a 70 kDa protein belonging to heat shock protein family which is abundantly produced in response to various forms of stress, such as toxic agents, oxidative stress, infection and heat shock [54]. Moreover, such family are responsible to protect cellular homeostatic processes from environmental and physiologic injuries via preserving structure of normal proteins [39]. It is well known that ethanol-triggered generation of ROS could suppress Hsp70 expression and intensifies oxidative damages [16]. Several in parallel studies exhibited that up-regulation of HSP70 protein in rats treated with various effective synthetic or natural compounds indicated protection of gastric mucosa against induced injuries by ethanol [21, 42, 55, 56]. Also our findings showed that administration of CNBP in the rats, induced significant up-regulation of Hsp70 protein levels in both reference and test groups (CNBP). Therefore, the up-regulation of HSP70 that was observed in the current study, suggested that the CNBP protected the gastric tissues via up-regulation of HSP70. Additionally, HSP70 are suggested to exert its cytoprotective activity through protecting mitochondria and interfering with stress-induced apoptotic program.

## Conclusions

The present study elucidated the anti-ulcer effect of CNBP against ethanol-induced gastric lesions. Acute toxicity test did not show any mortality or obvious sign of CNBP. The gastroprotective mechanism of CNBP might be suggested via increasing SOD, CAT activities, which in turn suppressed gastric acidity and prevented destruction of gastric mucus wall. Also there was notable reduction in MDA and PGE2 levels upon intake of the CNBP. In histological analysis, decrease of hemorrhagic mucosal region in gastric wall together with reduction or inhibition of edema and leukocytes infiltration of sub-mucosal layers was also observed. PAS staining reduction induced by ethanol was reversely increased by CNBP pre-treatment and also caused an increase in glycoprotein content. Immunohistochemistry analysis of gastric homogenate elicited critical role of Hsp70 up-regulation. The present study provided histological evidences on gastroprotective property of CNBP and also suggested that the compound could preserve of gastric mucus secretion and enhance antioxidant activities of CAT, SOD.

## Abbreviations

ALT: Alanine transaminase
AP: Alkaline phosphatase
AST: Aspartate transaminase
CAT: Catalase
CB: Conjugated bilirubin
CNBP: 2, 2′-[1, 2-cyclohexanediylbis (nitriloethylidyne)]bis(4-bromophenol)
FRAP: Ferric reducing antioxidant power
GGT: G-Glutaml transferase GGT
GWM: Gastric wall mucus
HSP70: Heat shock proteins 70
MDA: Malondialdehyde
MTT: 3-(4,5-dimethylthiazol-2-yl)-2,5-diphenyltetrazolium bromide
PGE_2_: Prostaglandins E_2_
SD: Sprague Dawley
SOD: Superoxide dismutase
TB: Total bilirubin
